# Prenatal Monitoring of Perinatal Pregnant Women and Fetus Based on a Smart Electronic Fetal Monitoring System

This article has been retracted.

**DOI:** 10.1155/2022/5073636

**Published:** 2022-11-18

**Authors:** Yu Sun, Su'e Jiang

**Affiliations:** Huai'an Maternal and Child Health Care Hospital, Huai'an 221006, China

## Abstract

The aim of the study is to study the prenatal monitoring of perinatal pregnant women based on a smart electronic fetal monitoring system. Through the comparative analysis of 230 pregnant women in maternal and child health care hospital who received fetal heart monitoring during the perinatal period and those who did not receive fetal heart monitoring during the perinatal period, cases of fetal distress, neonatal asphyxia, and cesarean section were observed in both groups. Results show that the incidences of fetal complications and cesarean sections in the experimental group were 16.36% and 36.82%, which was significantly higher than 4.50% and 17.50% in the control group(*p* < 0.05); the neonatal mild and severe asphyxia rates in the experimental group were 3.18% and 1.36%, which were significantly lower than 9.50% and 6.50% in the control group (*p* < 0.05). The experimental results show that the correct application of fetal heart rate monitoring in the perinatal period can aid in early detection and dealing with fetal distress and reduce the occurrence of various complications such as neonatal asphyxia. It is worthy to be popularized and applied in clinics.

## 1. Introduction

Fetal distress caused by intrauterine hypoxia is an important factor leading to fetal death. According to statistics, at least 30% of newborns born every year have cerebral palsy and 10% of patients with severe mental retardation are caused by fetal intrauterine hypoxia. The fetal heart is an organ that supplies oxygen and transports nutrients. It is controlled by the central nervous system of the brain and regulated by body fluids such as blood flow hormones (Figure 1). If there are problems, it can lead to fetal distress, growth retardation, even premature delivery, and dystocia [1]. However, these clinical features can be reflected from the changes of the fetal heart rate and uterine contractility (CTG) curve. CTG is a kind of monitor that describes the fetal heart rate and uterine contractile pressure of pregnant women and is also called a heart delivery force recorder. Different fetal heart contractions (CTG) have a complete set of different interpretation methods. The traditional interpretation method is to analyze the fetal heart contraction curve with the naked eye and experience. In recent years, the electronic fetal heart rate monitoring system has developed rapidly. With the introduction of computer-aided analysis of characteristics of the fetal heart rate cardiotocograph (CTG) curve and clinical parameters, fetal heart rate changes due to anemia or hypoxia can be detected early. Therefore, a smart electronic fetal monitoring system is of great significance for eugenics, early detection of fetal abnormalities, and prevention of fetal damage [2, 3]. At present, it is the most commonly used, sensitive, and effective monitoring method of fetal intrauterine conditions. Especially for the third trimester of pregnancy, effective fetal electronic monitoring can timely find the existence of fetal distress, and then through active and effective intervention, the incidence and mortality of various complications such as neonatal asphyxia can be significantly reduced.

## 2. Related Works

Gomez, O., pointed out through research that the fetus should be monitored after 32 weeks of pregnancy. On the one hand, it can ensure high security. On the other hand, it can minimize and avoid a series of adverse results caused by iatrogenic over prediction. [4]. Han, J., and others suggested that antenatal fetal monitoring should be initiated at 32–34 weeks of gestation. If pregnant women had high-risk factors such as diabetes, the start-up time should be advanced to 26–28 weeks. We chose the time to start fetal heart rate monitoring for pregnant women without complications at 36 weeks of pregnancy [5]. Khan, S. M., and others conducted a prenatal fetal heart monitoring on 780 pregnant women and screened 756 cases of the reactive type and 41 cases of the nonreactive type. The rate of reactive cesarean section was 25.1% (196/756), and the rate of nonreactive cesarean section was 61.0% (25/41) [6]. Amjad O. performed NST once a week for 1400 pregnant women after 36 weeks of pregnancy. The value of NST in predicting fetal condition was studied. The Apgar score of less than 7 was used as the judgment standard of neonatal asphyxia. The results showed that 18 cases (1.3%) of 1320 reactive types and 36 cases (45%) of 80 nonreactive types had neonatal asphyxia[7]. Huang, Q., and others proposed that fetal distress is when the fetal heart rate is more than 160 or less than 100 times per minute. Irregular fetal rate and fetal agitation are also manifestations of fetal hypoxia [8]. Johnston, J. C., and others believe that the application of Internet technology and short-range wireless transmission technology to the electronic fetal monitoring system has become a hot spot of research for current experts and scholars. The traditional fetal monitoring mode has also changed greatly, and the traditional mode of “arriving at the hospital after the disease” has begun to move toward the modern medical mode of “early prevention and early active diagnosis and treatment” [9]. Oweis, R. and others believe that the traditional fetal monitoring equipment can only be monitored in the hospital. The monitoring host is huge and bulky. Pregnant women have a baby and heavy body. For each prenatal examination, the patient needs to travel back and forth between home and the hospital, which brings great trouble to pregnant women [10]. When Pitts, D. S. and others found the development and application of wireless communication technology and Internet technology. Various portable wireless monitoring devices appear, such as portable fetal heart rate monitor, central monitoring station, and intelligent electronic fetal monitoring system [11].

## 3. Experimental Analysis

### 3.1. Data and Methods

#### 3.1.1. General Information

230 pregnant women in maternal and child health care hospital were selected to form the experimental group. They were 21 ∼ 39 years old, with an average of 26.6 ± 5.1 years old. The gestational weeks were 36 ∼ 42 weeks, with an average of 39.8 weeks. Among them, 170 cases were primipara and 60 cases were postmenopausal women; 190 cases were normal pregnancy and 30 cases were high-risk pregnancy. 200 parturients in the hospital with detailed records in the past were selected as the control group; they were 21–41 years old, with a mean of (25.5 ± 5.6) years old; the gestation week lasts 35 to 42 weeks, with an average of 39.5 weeks; among them, 154 cases were primipara and 46 cases were postmenopausal women; 172 cases were normal pregnancy and 28 cases were high-risk pregnancy. There were no significant differences in age, gestational period, and total pregnancy rate between the two groups (*p* > 0.05). The details are shown in Table 1 below.

#### 3.1.2. Method

When the pregnant woman is in the non-starvation state, the body position is taken as the semi-recumbent position or the left recumbent position. The ultrasonic Doppler probe is fixed at the position with the clearest fetal heart sound, and the uterine contraction probe is fixed at the two transverse fingers under the uterus to receive the signal. The fetus is monitored routinely for 20 minutes. In case of abnormality, it shall be extended to 30 ∼ 60 min and rechecked in time to eliminate the impact of fetal sleep, pregnant women's spirit, and other factors on the monitoring results. If the uterine orifice of pregnant women expands more than 2 cm, continuous monitoring shall be carried out [12], with a minimum time of 0.5 h and a maximum time of 7.5 h, and no sedatives shall be used. Non-stimulation test, oxytocin test, and uterine contraction test were carried out according to relevant standards.

*(1) NST Examination*. All pregnant women had routine NST examination once a week from the 36th week of pregnancy until delivery. The pregnant woman takes the semi-recumbent position and the ultrasonic probe is placed on the abdomen (fetal heart sound area) after coating the coupling agent, and fixed with an abdominal band. The paper feeding speed is set at 3 cm/min. While tracing the fetal heart rate, when the pregnant woman feels that fetal movement occurs, the fetal movement tracing button is pressed by hand to make a mark on the paper [12]. Continuous recording shall not be less than 20 min. If the fetal heart rate is 120–160 beats/min, the baseline rate rises to 15 beats/min or more, and the fetal movement is 2–4 or more, and each time lasts for more than 15s, it is a reactive type; if the abovementioned indicators are not met, the monitoring time shall be extended for 30–40 min, and the examiner shall gently push the abdomen of the pregnant woman to stimulate the fetus. If the abovementioned indicators can be met, it is still considered that NST has a response [13]. For those who fail to meet the above indicators, the nonreactive type can be judged only after monitoring for at least 40 min, the baseline variability is below 6bpm, there is no fetal movement, or there is fetal movement without fetal heart rate acceleration and the duration of acceleration amplitude is below the reactive type standard.

#### 3.1.3. Observation Index

Cases of fetal complications, neonatal asphyxia, and cesarean delivery have been reported. Diagnostic criteria of fetal distress: when the fetal heart rate is ≤ 120 beats/min or ≥160 beats/min, it indicates that the fetus has hypoxia; in terms of fetal movement, at first, fetal movement was frequent, and then fetal movement decreased or disappeared; amniotic fluid: those with grade II ∼ III fecal contamination; and in terms of umbilical cord, the S/D ratio of umbilical cord blood flow ≥2.6. Diagnostic criteria of neonatal asphyxia: mild asphyxia with an Apgar score of 4 ∼ 7 at 1 minute of birth; an Apgar score of 0 ∼ 3 at 1 min of birth is severe asphyxia [12].

### 3.2. Result Analysis

According to statistics, the fetal complications and cesarean section rates in the experimental group were 16.38% (36/220) and 36.81% (82/220), which is significantly higher than 5.40% (9/200) and 17.60% (35/200) (*P* < 0.05) in the control group. The mild and severe asphyxia of newborns in the experimental group were observed 3.28% (7/220) and 1.43% (3/220), respectively, significantly lower than 9.60% (19/200)) and 6.50% (13/200) of the control group (*p* < 0.05). See Table 2.

Relationship between NST examination results and neonatal asphyxia: there were 190 cases of the NST reactive type, including 10 cases of mild neonatal asphyxia, accounting for 1.18%. There were 49 cases of the NST unresponsive type, including 18 cases of neonatal mild asphyxia, accounting for 36.73%, 2 cases of severe asphyxia, accounting for 4.09%, and 20 cases of asphyxia, accounting for 40.82%. There was a very significant difference between the two groups (*p* < 0.01).  Figure 2 shows the specific experimental results.

## 4. Discussion

According to the existing research results, neonatal asphyxia is still a very important cause of neonatal death and disability. The latest foreign reports show that its incidence is 5% ∼ 6%, while in China, it also has an incidence of 4.7% ∼ 8.9%. According to the survey results of 18 cities in China, asphyxia and its complications account for 33.5% of the death causes of newborns. It is generally believed that the occurrence of neonatal asphyxia and complications is a continuation of fetal intrauterine distress, which indicates that in the clinical process, we should study the causes of fetal intrauterine distress and deal with it timely and effectively. Fetal intrauterine distress generally refers to a series of clinical manifestations caused by fetal circulatory hypoxia in the uterus, which is an important complication during delivery; in terms of clinical manifestations, it is mainly the abnormal fetal heart rate and decreased or disappeared fetal movement. In the actual clinical work [14], researchers generally take the abnormality of fetal heart rate and meconium pollution as the main diagnostic criteria, this requires careful monitoring of changes in the fetal heart rate. This is caused by fetal hypoxia, the peristalsis of the intestine shows a certain hyperactivity, while the anal sphincter is relaxed, and the meconium is discharged into the amniotic fluid, causing pollution. The fetus inhales the meconium into the trachea, aggravating the hypoxia. This requires medical workers to clear the respiratory tract after the delivery of the fetus and ensure the smoothness of the respiratory tract, which has become the primary task of rescuing neonatal asphyxia. In the process of observation, if there is serious meconium pollution, they can choose to terminate the pregnancy immediately to prevent asphyxia and other complications. Various factors of blood gas exchange between the mother and fetus can cause fetal distress. Various factors of decreasing blood oxygen saturation can lead to neonatal asphyxia, which can occur at any stage of pregnancy, but most of them occur after the beginning of labor. If there is severe hypoxia in this process, it may cause fetal death in uterus [14].

Changes in fetal heartbeat are regulated by the fetal central nervous system, and fetal heartbeat acceleration and fetal movement are considered to be the circulatory system's response to fetal movement. It is believed that stimulating fetal movement causes the fetal heartbeat to accelerate through the central nervous system, such as the cerebral circulation. Therefore, fetal heart monitoring is the monitoring of the cardiac regulation function of the fetal central nervous system. In order to correctly respond to the health status of the fetal central nervous system, it can be used to judge whether the fetus has intrauterine hypoxia and its severity, and take effective measures according to specific conditions, such as intrauterine resuscitation or termination of pregnancy, which can prevent fetal acidosis and secondary damage to fetal heart, brain, liver, kidney and other tissues and cells; improve the prognosis of the fetus; improve the occurrence of various complications and sequelae of the newborn; and improve the quality of life of the newborn. In the process of monitoring, the midwife should closely observe the changes of fetal heart rate and uterine contraction pressure, make various relevant necessary records, and adjust the probe position in time according to the situation, so that the fetal heart signal transmission is the clearest and most convenient, and the results obtained are the most authentic and credible. It also requires obstetricians to have a clear and full understanding of various changes of fetal heart rate, make sufficient preparations before fetal delivery, correctly deal with each stage of labor, and actively prevent the occurrence of premature birth and low birth weight infants, which play a positive role in reducing the occurrence of neonatal asphyxia.

### 4.1. Algorithm for Deriving the Fetal Heart Rate Curve

#### 4.1.1. Analysis of the Fetal Heart Rate Baseline Extraction Algorithm

Baseline FHR is defined as the average fetal heart rate over 10 minutes in the absence of fetal movement or uterine contractions as the fetal heart rate base (e.g., FHR base). The fetal heart rate graph recorded on the monitor is a fluctuating band-like curve. According to the baseline fetal heart rate, the fetal heart rate curve can be divided into three types: tachycardia, normal, and bradycardia. The classification framework is shown in Table 3.

The fetal heart rate is susceptible to stimuli such as fetal movement, contractions, and palpation, and will temporarily accelerate and decelerate (for 10–20 s) before returning to the baseline. Because it is easy to update the fetal base and body time, it is necessary to accurately calculate the heart rate throughout the fetal period [15].

Based on the clinical characteristics of the fetal heart rate, a method for estimating baseline fetal heart rate was developed in this paper. The main idea of the algorithm is as follows: (1) First read the fetal heart rate data, delete the fetal heart rate data (data other than 90–200 times/min), analyze the remaining data with histogram, and record the fetal heart rate and histogram with FHR, as the base value, accounts for the largest proportion of the remaining data. (2) Taking the baseline as the reference point, the fetal heart curve is smoothed and filtered. (3) The fetal heart rate curve varies greatly, and it is not recommended to use the smoothening algorithm alone. Therefore, the steep part of the change must be corrected and filtered after the threshold is set. (4) After four thresholds of correction and repeated processing, a relatively uniform baseline fetal heart rate can be obtained.

When obtaining the position of reference point through histogram analysis, first the fetal instantaneous heart rate from BPM to time domain unit (fetal cardiac cycle) is converted to facilitate the calculation and screening of the fetal heart rate data. For example, the selected fetal heart rate range is 90bpm-200bpm and the time domain is 300ms-600 ms. The fetal heart rate reference point can be reflected by finding a relatively concentrated fetal heart cycle in a sampling point through the histogram. As shown in Figure 3, the position and size of the reference point (inverted triangle identification) can be obtained by intuitive observation.

The smoothening filtering adopts forward and backward smoothening at the same time. The obtained reference point is used as the reference point *B*_0_ for the smooth filtering of the fetal heart rate, and the filtering processing is carried out on the basis of *B*_0_. The forward and backward filtering formulas are as follows:

Initial position: *B*_0_=0.975*B*_0_+0.025*B*_*i*_

Forward filtering: *B*_*i*_=0.965*B*_*i*+1_+0.035*B*_*i*_

Backward filtering: *B*_*i*_=0.965*B*_*i*−1_+0.035*B*_*i*_

If the fetal heart rate fluctuates greatly, smoothening is not recommended, and the part with large fluctuation needs to be corrected. The process of correcting the algorithm is to preset an upper and lower threshold. When the fetal heart rate data are greater than the upper threshold of the baseline, the current fetal heart rate value is replaced. According to the set threshold, the position and size of the point to be replaced can be found. Similarly, when the fetal heart rate data are less than the lower threshold of the flow baseline [16], it is replaced in the same way. The closed value parameter settings of three iterations are shown in Table 4.

As shown in Figure 4, the baseline of fetal heart rate during the whole monitoring process is obtained. The thin line with large fluctuation is the instantaneous rate curve of the fetal heart rate, and the thick line more stability and smoothness is the baseline of the fetal heart rate.

#### 4.1.2. Analysis of FHR Acceleration and FHR Deceleration Algorithms

Fetal heart rate acceleration is defined as a temporary increase in fetal heart rate at baseline, the fetus is not less than twice within 20 minutes after the beginning of the experiment, and the instantaneous rate is greater than the baseline of fetal heart rate by more than 15bpm for more than 15 s. In the process of fetal development, acceleration begins to appear about 18 weeks of pregnancy, and the improvement of acceleration mechanism is after 28–29 weeks. Therefore, acceleration is an important physiological phenomenon in the third trimester of pregnancy and an index to judge the health and safety of the fetus in the womb. There are two main types of acceleration: periodic acceleration and aperiodic acceleration. Nonperiodic acceleration occurs with fetal movement, internal diagnosis, or abdominal palpation. Periodic contractions accompany uterine contractions, with an increase in the fetal heart rate occurring in tandem with the contractions. Based on the fetal heart rate definition, an algorithm was developed to accelerate the fetal heart rate. The basic process is as follows: (1) obtain the baseline of fetal heart rate and detect the instantaneous FHR value of each sampling point. (2) Find the data greater than 10bpm of FHR baseline value, search the maximum value in the next minute, and record the peak value and occurrence time. (3) Then, search for points 3 BPM larger than the baseline value in 55s forward and backward respectively. (4) In the third step, search the FHR minimum value point of the corresponding time range, and record the occurrence time as the starting point and ending point [17].

The definition of fetal heart rate deceleration is the temporary deceleration of fetal heart rate accompanied by uterine contraction. It can be divided into periodic deceleration and aperiodic deceleration according to the occurrence time, shape, and continuous length. At present, most of them still use Edward Hon's method to classify, record the fetal heart rate and uterine contraction curve for 40–60 minutes, and then see whether the deceleration pattern of each fetal heart rate is basically the same and whether the deceleration waveform has a certain relationship with the uterine contraction waveform. Periodic deceleration is judged according to the time-position relationship between the fetal heart rate curve and uterine contraction. It is divided into early deceleration, late deceleration, and variable deceleration. Their clinical manifestations are as follows: (1) Early deceleration generally occurs in the later stage of the first stage of labor. Uterine contraction is caused by fetal head compression and is not changed by the pregnant women's body position or oxygen inhalation. (2) Mutation decelerates, suggesting umbilical cord compression. (3) The classification range of late deceleration, placental dysfunction, and fetal hypoxia is shown in Table 5.

The idea and process of deceleration detection algorithm is similar to that of acceleration algorithm: (1) obtain the baseline of fetal heart rate and detect the instantaneous FHR value of each sampling point. (2) Find the data less than 20bpm of FHR baseline value, and search the minimum value, marked trough value and occurrence time in the next minute. (3) Then, search for points 3 BPM smaller than the baseline value in 55s forward and backward, respectively. (4) Find the point that meets the conditions (FHR in the corresponding range is the fetal heart rate deceleration event) and mark the decline amplitude and occurrence time. The actual detection effect is shown in Figure 5. The acceleration event points detected above the baseline are marked with “*∗*“, and the deceleration event points detected below the baseline are marked with “+“, so that the number and time of fetal heart rate acceleration and deceleration can be obtained.

## 5. Conclusion

In this study, the incidence of fetal distress and cesarean section rate in the experimental group were significantly higher than those in the control group (*p* < 0.05). The rates of mild and severe neonatal asphyxia in the experimental group were significantly lower than those in the control group (*p* < 0.05). To sum up, the correct application of fetal heart rate monitoring in the perinatal period can early detect and deal with fetal distress and reduce the occurrence of various complications such as neonatal asphyxia, which is worthy of popularization and application in clinics. The smart electronic fetal monitoring system realizes intelligent monitoring through Internet of things technology, Internet platform, and portable sensor equipment, and uploads the monitoring data to the cloud. Doctors and pregnant women interact through the intelligent maternal and infant care platform based on the Internet of things and cloud platform. Doctors can timely understand the health status of pregnant women and fetuses and remotely guide them to carry out corresponding operations. Pregnant women can enjoy the same supervision as in the hospital anytime and anywhere. The whole maternal and infant monitoring system constitutes a network system with monitoring, analysis, and feedback functions, which realizes smart monitoring anytime and anywhere, and reduces the pain of patients running between families and hospitals. In terms of fetal heart rate detection, obstetric experts and large sample clinical data need to be tested repeatedly to optimize and improve the recognition algorithm of relevant parameters of fetal heart rate contraction curve, so as to improve its accuracy and reliability.

## Figures and Tables

**Figure 1:** Fetal detection system.

**Figure 2:** Relationship between NST examination results and neonatal asphyxia.

**Figure 3:** Analysis of the fetal heart rate baseline by a histogram method.

**Figure 4:** Baseline detection and analysis of fetal heart rate.

**Figure 5:** Analysis of fetal heart rate deceleration and deceleration detection.

**Table 1:** Experimental object situation table.

	Age	Gestational week (weeks)	Primipara	Normal pregnancy	High-risk pregnancy
Experience group	26.6 ± 5.1	39.8	170	190	30
Control group	25.5 ± 5.6	39.8	154	46	172

**Table 2:** Comparison of fetal complications and cesarean section between the two groups (N%).

Group	Number of cases	Fetal distress	Mild neonatal asphyxia	Severe neonatal asphyxia	Cesarean section
Experience group	230	36 (16.38)	7 (3.28)	3 (1.43)	82 (36.81)
Control group	200	9 (5.40)	20 (9.60)	13 (6.50)	34 (17.60)
*p* Value		<0.05	<0.05	<0.05	<0.05

**Table 3:** Baseline classification of the fetal heart rate.

Classification		Variation range (times/minute)
Normal		120–160

Tachycardia	Light	161–180
	Severe	Above 180

Bradycardia	Light	100–119
	Severe	Below 99

**Table 4:** Parameter setting of baseline correction threshold of the fetal heart rate.

Number of iterations	Upper threshold (bpm)	Lower threshold (bpm)
1	25	20
2	20	15
3	10	10

**Table 5:** Types of fetal heart rate deceleration.

	Decrease of fetal heart rate	Lag time	Deceleration duration
Get up early and slow down	[l5, 50] bpm	≤15 s	60–70 s
Late deceleration	[15, 30] bpm	[30, 60] s	60–70 s
Mutation deceleration	≥15 bpm	Uncertain	15–20 s

## Data Availability

The data that support the findings of this study are available from the corresponding author upon request.
